# Macular Hole Detection Using a New Hybrid Method: Using Multilevel Thresholding and Derivation on Optical Coherence Tomographic Images

**DOI:** 10.1155/2021/6904217

**Published:** 2021-12-22

**Authors:** Sahand Shahalinejad, Reza Seifi Majdar

**Affiliations:** ^1^Department of Electrical and Computer Engineering, Urmia Higher Education Institute, Urmia, Iran; ^2^Department of Electrical Engineering, Ardabil Branch, Islamic Azad University, Ardabil, Iran

## Abstract

Optical coherence tomography (OCT) is a noninvasive imaging test. OCT imaging is analogous to ultrasound imaging, except that it uses light instead of sound. In this type of image, microscopic quality intratissue images are provided. In addition, fast and direct imaging of tissue morphology and reproducibility of results are the advantages of this imaging. Macular holes are a common eye disease that leads to visual impairment. The macular perforation is a rupture in the central part of the retina that, if left untreated, can lead to vision loss. A novel method for detecting macular holes using OCT images based on multilevel thresholding and derivation is proposed in this paper. This is a multistep method, which consists of segmentation, feature extraction, and feature selection. A combination of thresholding and derivation is used to diagnose the macular hole. After feature extraction, the features with useful information are selected and finally the output image of the macular hole is obtained. An open-access data set of 200 images with the size of 224 × 224 pixels from Sankara Nethralaya (SN) Eye Hospital, Chennai, India, is used in the experiments. Experimental results show better-diagnosing results than some recent diagnosing methods.

## 1. Introduction

Optical coherence tomography (OCT) is a fundamentally new type of optical imaging modality. OCT performs high-resolution, cross-sectional tomographic imaging of the internal microstructure in materials and biologic systems by measuring backscattered or backreflected light. OCT images are two-dimensional data sets that represent the optical backscattering in a cross-sectional plane through the tissue. Image resolutions of 1 to 15 *μ*m can achieve one to two orders of magnitude higher than conventional ultrasound. Imaging can be performed in situ and in real-time [1]. The unique features of this technology enable a broad range of research studies and clinical applications [2]. Mendes and Abrah 2019 provide an overview of OCT technology, its background, and its potential biomedical and clinical applications. OCT, imaging the internal cross-sectional microstructure of tissues using measurements of optical backscattering or backreflection, was first demonstrated in 1991. OCT imaging was performed in vitro in the human retina and atherosclerotic plaque as examples of imaging in transparent, weakly scattering media and nontransparent, highly scattering media. OCT was initially applied for imaging in the eye and to date. OCT has had the largest clinical impact in ophthalmology. The first in vivo tomograms of the human optic disc and macula were demonstrated in 1993 [3]. OCT enables the noncontact, noninvasive imaging of the anterior eye as well as imaging of morphologic features of the human retina including the fovea and optic disc. Numerous clinical studies have been performed by many groups in the last several years. More recently, advances in OCT technology have made it possible to image nontransparent tissues, thus enabling OCT to be applied in a wide range of medical specialties. Imaging depth is limited by optical attenuation from tissue scattering and absorption. However, imaging up to 2 to 3 mm deep can be achieved in most tissues. This is the same scale as that typically imaged by conventional biopsy and histology. Although imaging depths are not as deep as with ultrasound, the resolution of OCT is more than 10 to 100 times finer than the standard clinical ultrasound [4]. OCT has been applied in vitro to image arterial pathology and can differentiate plaque morphologies. Imaging studies have also been performed in vitro to investigate applications in dermatology, gastroenterology, urology, gynecology, surgery, neurosurgery, and rheumatology. OCT has also been applied in vivo to image developing biologic specimens for applications in developmental biology. OCT is of interest because it allows repeated imaging of developing morphology without the need to sacrifice specimens. Numerous developments in OCT technology have also been made. High-speed real-time OCT imaging has been demonstrated with acquisition rates of several frames per second. High-resolution and ultrahigh-resolution OCT imaging has been demonstrated using novel laser light sources, and axial resolutions as high as 1 *μ*m have been achieved. Cellular level OCT imaging has recently been demonstrated in developmental biology specimens. CT has been interfaced with catheters, endoscopes, and laparoscopes which permit internal body imaging. Catheter and endoscope OCT imaging of the gastrointestinal, pulmonary, and urinary tracts as well as arterial imaging has been demonstrated in vivo in an animal model. In many cases, the disease is examined only superficially (without considering the complete characteristics involved in the disease). Many research groups are currently performing preliminary clinical studies.

The macular located in the middle of the retina is where most of the cone cells accumulate. A small depression in the middle of the macular called FOA has the largest cone cell. The macular is responsible for central vision, hue vision, and accurate detail recognition. The cylindrical cells are located in the peripheral part of the retina (around the retina) and allow night vision and the movement of objects around. The partial or complete absence of the macular sensory membrane is called macular perforation. The macular hole may be of an unknown and age-related cause (age-related macular hole) or maybe caused by trauma to the eye. The age-related type of the disease is most prevalent in older women in the seventh decade of life. The OCT images of normal and abnormal macular are shown in Figure 1.

## 2. Related Works

In connection with macular pathologies, we face some harms such as macular edema, age-related macular degeneration (AMD), macular edema, central serous retinopathy (CSR), and macular hole (MH) [5–7]. Macular holes lead to low vision and blindness, which can lead to retinal holes due to overuse of fovea [8]. The disease is more likely to occur in people over 40 years of age [9].

Early diagnosis of the disease will help a lot in its treatment because if the disease progresses little, it can be treated with the help of medicine or surgery. Therefore, knowing the characteristics of the hole such as shape, size, width, diameter, and length can be very effective [10–12]. OCT image is an effective tool to diagnose the condition of an MH [13–15].

The OCT is an applicable tool to diagnose the retina pathologies, which can visualize the 3D shape and structure of the retina without physical contact [16–18]. The high-resolution OCT images of the retina usually have speckle noise and shadows caused by retinal blood vessels and other abnormalities on retina, which are challenges in the segmentation process [19–26].

Because the disease can cause irreparable damage if misdiagnosed by algorithms, manual segmentation has always been a priority, but our algorithm ignores the use of this method with a very low error coefficient to detect the macular hole [27–32] Even in some cases, the correct diagnosis of a disease depends on several studies. Nevertheless, the need for fully automatic diagnostic methods for retinal pathology is now felt.

One of the important applications of OCT images is to detect MH (Figure 1). Therefore, the researchers want to propose full automated, novel, and trustfully methods for MH diagnosis and segmentation [33, 34]. New research studies in this area seek to cover each other to reduce each other's shortcomings and to make them acceptable methods by experts. The valuable information and features provided by OCT images can help researchers develop more valuable segmentation and automated diagnostic techniques to help patients lead better lives [35, 36].

In [37], a fully automatic method to identify the main layers of the retinal that delimits the retinal area is proposed. Therefore, an active contour-based model is used to segment the main retinal boundaries. This method uses the horizontal placement information of these layers and their relative location on the images to restrict the search space. A new OCT-based method to investigate epiretinal membrane (ERM) pathology in human eyes is proposed by Gonz'alez-L'opez et al. [38]. The new approach assesses automatically the ERM thickness and the space between the epiretinal membrane (ERM) and the retina surface. The adjusted mean arc length (AMAL) for segmenting OCT images for macular pathology is being used for segmenting OCT images for macular pathology [39]. This metric is used for automated OCT segmentation. In recent years, a segmentation method based on feature extraction using SFTA-based histological analysis has been introduced by Keller et al. [40]. In this research, a graph-based segmentation is used to find the layers of retina. The 3D level set segmentation approach based on the level set method can used to accurate segmentation of the MH [41]. This method is fully automatic and shows robust results in a variety of conditions. A novel layer guided convolutional neural network (LGCNN) is proposed by Nasrulloh et al. [42] to identify the common types of macular pathologies and normal retina. In this method, the retinal layer segmentation maps are generated by an efficient segmentation network, which can determine two lesion-related retinal layers associated with the meaningful retinal lesions. Then, two subnetworks in LGCNN integrate the information of these layers. Consequently, by focusing on the significant lesion-related layer regions, LGCNN can effectively modify OCT classification. Huang et al. [43] proposed a multi-instance multilabel-based lesions recognition method to detect and recognize simultaneously multiple lesions. The proposed method consists of the segmentation based on the different lesions and feature extraction and constructs multilabel detectors and recognizes the region of interests. A unique joint model that combines multiple information is proposed for retinal segmenting using OCT images [44]. A multimodal multiresolution graph-based method is proposed for internal limiting membrane segmentation within OCT images [45]. A hybrid method using multilevel thresholding and derivation on optical coherence tomographic images was proposed for automated detection [46, 47].

In this paper, a new combination is proposed to obtain more information for macular hole diagnostic. This is a multistep method, which consists of segmentation, feature extraction, and feature selection. A combination of thresholding and derivation is used to diagnose the macular hole. After feature extraction, the features with useful information are selected and finally the output image of the macular hole is obtained. The main contributions of the proposed method are (1) high sensitivity in the various OCT images, (2) better accuracy and reliability than the conventional methods, and (3) short processing time.

The remaining parts of this paper are organized as follows: In Section 3, the mentioned proposed method is introduced. Experiments and results can be found in Section 4. Comparison with some recent methods is demonstrated in Section 5, and the conclusion is given in Section 6.

## 3. Proposed Methods

The block diagram of the proposed method is shown in Figure 2. The proposed method consists of multiple steps. The preprocessing step is usually used before the main image analysis and data extraction, and its purpose is to obtain an accurate image that removes annoying data from the image. In medical imaging, major disorders are observed, including noise due to high-frequency reception, different brightness in the field, and problems due to distant orientation. For this reason, preprocessors are applied to all images taken from a device. For this reason, these processes are usually device dependent and must be fast and efficient. Photogrammetric methods are used when the spatial or luminous properties of the noise are known. In this paper, we used an adaptive filter to remove noise from OCT images. In the next step, the proposed algorithm is implemented on the images, and images have been qualitatively improved; therefore, their characteristics must be determined and extracted. Most image data may be subdivided into enclosed areas, dots, and lines. To identify objects, they must be able to distinguish them from the context. It is usually best to convert the gray spectrum image to a binary image (black and white). Techniques such as image splitting and edge recognition work best on binary images but are sometimes applied to images in the gray or color spectrum. The purpose of feature extraction is to extract features that are directly related to the output. After this step, the extracted features with basic information are selected and finally the output image is obtained.

In the proposed method block diagram (Figure 2), a combination of thresholding and derivation is used for diagnosis. This method has been implemented with special emphasis on FOA depression and image features in this area, and finally a suitable segmentation has been used to distinguish this disease from other diseases and the rate of disease progression. Edge as the location of changes in lighting levels, the range of these changes should also be considered to decide on the presence of the edge and its exact location. In this case, if the edges of an image are exposed, the location of all the prominent and opaque objects in the image is determined. As a result, the use of an accurate edge detector directly helps to increase the feature recognition rate and the ability to accurately segment the image. The vector *f* (*x*, *y*) represents the maximum rate of change of brightness.

(1) $$\begin{array}{c} f\left(x\right)=\frac{I_{r}-I_{\ell }}{2}\left(\text{erf}\left(\frac{x}{\sqrt{2}\sigma }\right)+2\right)+I_{\ell }. \end{array}$$

Outset of edge (*I*_1_) and end of edge (*I*_2_) are defined in the following equation:

(2) $$\begin{array}{c} L\left(x\right)=-1\cdot I\left(x-1\right)+0\cdot I\left(x\right)+1\cdot I\left(x+1\right), \end{array}$$

(3) $$\begin{array}{c} L_{x}=\left[\begin{array}{ccc} \text{0} & -1\\ +2 & \text{0} & -2\\ +1 & \text{0} & -1 \end{array}\right]L\text{ and }L_{y}=\left[\begin{array}{ccc} +2 & +1\\ \text{0} & \text{0} & \text{0}\\ -1 & -1 & -1 \end{array}\right]L, \end{array}$$

(4) $$\begin{array}{c} \left|\nabla L\right|=\sqrt{L_{x}^{2}+L_{y}^{2}},\theta =\arg\;\tan\;2\left(L_{y},L_{x}\right). \end{array}$$

On the other hand, when the multilevel thresholding method is applied, it converts the gray level into a binary code. The key point in this method is to select the threshold value (or threshold values for the case where several levels are desired). Most images include objects with a uniform brightness level on a background with different brightness levels. For such images, brightness is a distinguishing feature that can separate the object from the background. Another way to choose the value of the threshold of light is to place the threshold value equal to the minimum point of the histogram between the two peaks.

## 4. Experiments and Results

### 4.1. Data Set

In this paper, we use the open-access database collected by Lakshminarayanan et al. 2019 [48]. This database includes more than 500 high-resolution OCT images of different pathological conditions. A raster scan protocol with a 2 mm scan length was used to obtain these images. The size of these images is 512 × 1024 pixels and took using a Cirrus HD-OCT machine (Carl Zeiss Meditec, Inc., Dublin, CA) at Sankara Nethralaya (SN) Eye Hospital, Chennai, India. In each volumetric scan, a fovea-centered image was selected by an experienced clinical optometrist (MKP). The axial resolution was 5 *μ*m, and the transverse resolution was 15 *μ*m (in tissue). The images were then resized to a 224 × 224 pixel size. The pathological conditions were determined by clinicians, and the labeling process was done by retinal clinical experts at SN hospital. Progressive stages and macular degeneration are given. This wide range of stages, less severe, medium severe, and more severe stages, in each disease would be ideal for the researchers; therefore, they can test their proposed method in various scenarios. MH OCT images are the main category of the database, and we used several images of MH cases.

### 4.2. Initialization

The raw data were used separately, in the mentioned method using MATLAB 2019a software to identify macular hole; in the first stage, OCT images were collected as input, with background uniformity and improved image resolution, under preprocessing. In the second stage, identification was performed using the segmentation method and the desired points were examined from the image. In the third and final step, a new hybrid method is implemented on the images. To implement the simulated results, Corei7 CPU, GeForce 7900GTX graphics processing unit, and 16 GB of memory were used.

### 4.3. Experiments

In this part, the implementation results of the proposed method on OCT images provided by Lakshminarayanan et al. [48] are presented. The image derivation is an important step in many image-processing algorithms. The simplest case may involve applying one algorithm. More complex cases include more accurate margin detection algorithms or applying several separable models, given that time processing is also important. Using two methods of thresholding and derivation, we introduced a new and more efficient method than other methods (Figure 3). In the recognition of surfaces, the most important features can be extracted from the surfaces (including corners and lines). The output of the process is a set of parts whose community includes the whole image or a set of lines extracted from the image. Each pixel in each section is similar in which it has specific properties such as hue, brightness, or texture. Adjacent sections are considered different from each other according to the mentioned features. By recognizing the pixels in the image, considering the existence of valuable and important information in the image, a segmentation algorithm was used in which each pixel is assigned a label so that pixels with the same label have similar properties These features must have properties so that with a set of these features, each image can be described uniquely in order to identify the identity of an image from the patterns of that image. Mean sensitivity and mean accuracy for 12 sample OCT images are shown in Table 1.

The accuracy is computed by comparing the automated results with the ophthalmologist's diagnosis opinions. The proposed algorithm helps the ophthalmologist to educate the patient about the progression of the disease. This algorithm can aid the ophthalmologist by analysing the huge number of samples in a short time and presenting only the samples exhibiting features of diseases. An automated pre-exclusion of normal cases might help to improve the program's efﬁciency. In future work, we consider to improve the accuracy in the detection of macular hole. The results of applying the proposed algorithm are clearly shown on the images at each stage of processing.

## 5. Comparison

In order to compare the results of our proposed method with some recent segmentation methods, we compare it with SVM, KNN, Navie Bayes, Decision Tree, MS-LGDF, and CMF [49]. SVM, KNN, Navie Bayes, and Decision Tree are four traditional segmentation methods; MS-LGDF is a segmentation method based on the local Gaussian distribution fitting (LGDF) energy functional which can collect various macular hole measurements. The segmentation results such as accuracy, sensitivity, Jaccard index, and DSC are shown and compared in Table 2.

According to the comparison, it can be concluded that the proposed method is much better than the other methods. Image segmentation methods are of two main categories: border-based logic and area-based logic, and each of them it is divided into several techniques [50]. The output of a process is a set of sections whose assembly comprises the entire image or a set of lines extracted from the image [49]. Each pixel in each section is similar in which it has specific properties such as color, brightness, or texture. Adjacent sections are considered different from each other according to the mentioned features [51, 52].

In traditional methods, due to the complexity of the surface of the algorithms used, the accuracy was always low, the sensitivity was at the lowest level, and the long data processing time was clearly visible [52]. Image fragmentation has been done in areas such as computer vision and image processing, and due to its wide and wide application, it has suitable research fields. Despite the complexity of the algorithm, fragmentation has high accuracy and sensitivity and on the other hand fewer data processing time than traditional methods. The success of this research can be seen in other areas as well such as medicine. Remote and image retrieval is crucial, which helps to save, maintain, and protect human life [53].

The run times of the proposed combination method and other compared methods are tabulated in Table 3. The experiments were conducted on a computer with an Intel Corei7 CPU and 16 GB RAM running Windows 7 64Bit operating system. In addition, MATLAB version 2019a is used to obtain the computational times. As can be observed, the run time of the proposed method is better than that of the competition methods.

## 6. Conclusions

In this paper, we proposed an automatic and powerful method to segment OCT images to detect macular holes. This is a multistep method, which consists of segmentation, feature extraction, and feature selection. A combination of thresholding and derivation was used to diagnose the macular hole. After feature extraction, the features with useful information were selected and finally the output image of the macular hole was obtained. The proposed method was evaluated on an open-access data set from Sankara Nethralaya (SN) Eye Hospital, Chennai, India. Comparison with some state-of-the-art MH segmentation methods reveals the robustness of the proposed method. In the future, we want to develop this method for 3D segmentation and measurements.

## Figures and Tables

**Figure 1:** Samples macular images.

**Figure 2:** Macular hole detection block diagram.

**Figure 3:** Macular hole detection by the proposed method.

**Table 1:** Results by applying the proposed algorithm to the OCT images.

Experiment	Mean sensitivity (%)	Mean accuracy (%)
Image 1	87.56	97.25
Image 2	86.65	98.76
Image 3	88.87	96.98
Image 4	89.20	97.75
Image 5	87.12	98.15
Image 6	89.32	96.99
Image 7	88.59	96.50
Image 8	86.75	94.20
Image 9	89.99	98.81
Image 10	88.22	97.98
Image 11	87.70	96.93
Image 12	86.13	98.82

**Table 2:** Comparison between the proposed method and the other methods.

Image	Accuracy	Sensitivity	Jaccard index	DSC
SVM	80.5	79.2	65.3	78.2
KNN	75.7	72.4	63.8	73.1
Navie Bayes	78.4	78.2	64.2	74.2
Decision Tree	69.6	67.5	62.2	66.3
MS-LGDF	96.2	84.3	75.1	83.2
CMF	94.4	67.5	63.2	75.4
The proposed method	**97.5**	**88.3**	**78.5**	**85.3**

**Table 3:** Average run time comparison between the proposed method and some recent segmentation methods.

Methods	SVM	KNN	Navie Bayes	Decision Tree	MS-LGDF	CMF	Proposed method
Average run time (s)	68	72	59	70	89	86	54

## Data Availability

All data used in the database are valid.
